# The Correlation between Type 2 Diabetes and Fat Fraction in Liver and Pancreas: A Study using MR Dixon Technique

**DOI:** 10.1155/2022/7073647

**Published:** 2022-12-30

**Authors:** Yonghong Zheng, Shengsheng Yang, Xianyuan Chen, Jieqin Lv, Jiawei Su, Shun Yu

**Affiliations:** ^1^Shengli Clinical Medical College of Fujian Medical University, Fujian, Fuzhou, China; ^2^Department of Radiology, Fujian Provincial Hospital, Fujian, Fuzhou, China

## Abstract

**Objective:**

The increased obesity results in ectopic fat deposits in liver and pancreas, which will affect insulin resistance and elevated plasma glucose with type 2 diabetes. To assess the relationship between obesity and ectopic fat deposits and diabetes, this study used the MR Dixon method for the quantification of liver and pancreas fat fraction (FF) in type 2 diabetes mellitus (T2DM) patients and healthy controls.

**Methods:**

The FF of whole liver (FFWL) and pancreas (FFWP), the maximum diameters of the pancreas, the abdominal subcutaneous adipose area (SAT), the visceral adipose tissue area (VAT), and the total abdominal adipose tissue area (TAT) were measured for 157 subjects using the MR Dixon data. Four groups were established on the basis of BMI value. For statistics, intra- and intergroup comparisons were made by employing independent sample *t*-test.

**Results:**

FFWL, FFWP, and VAT varied significantly between T2DM (BMI < 25) and control group (BMI < 25), T2DM (BMI ≥ 25) and control group (BMI ≥ 25), T2DM (BMI < 25) and T2DM (BMI ≥ 25) (all *P* < 0.05). The FF of pancreas tail, SAT, and TAT varied significantly between control group (BMI < 25) and control group (BMI ≥ 25) (*P* < 0.05). FFWP and the FF of pancreas tail varied significantly between T2DM and normal volunteers (*P* < 0.05), with normal or mild liver fat content.

**Conclusion:**

The tissue FF, which has a close relationship with T2DM, can be assessed by the MR Dixon technique. T2DM patients should pay attention to tissue fat content regardless of BMI values.

## 1. Introduction

Obesity increases the amount of free fatty acids in the body. When normal adipose tissue cannot withstand excess fatty acids, fat accumulates into nonadipose tissue, such as liver and pancreas, resulting in ectopic fat deposits [1]. Previous studies [1–3] demonstrated that such ectopic fatty infiltration in the liver produces lipotoxic substances, and the high-fat concentration in liver among diabetic patients affects insulin resistance, plasma glucose, and metabolic control; fat deposit can also cause anatomical changes and abnormal secretion functions of the pancreas, leading to insulin resistance and blood sugar increase in the body. There is a close relationship between obesity and lipid metabolism disorders and diabetes, and thus, tissue fat quantification technique is highly required in clinical practice.

Liver and pancreas biopsies is considered as the gold standard for tissue fat quantification. However, performing lipid quantification through biopsy has some disadvantages. For example, such an invasive method may cause bleeding and infection. For another, biopsy only takes a small piece of the tissue for fat content measurement that cannot reflect the condition of the whole target tissue. Further, the pancreas is a peritoneal organ, easily interfered by other organs and the intestinal gas in the abdominal cavity during biopsy. All the abovementioned demerits limit the clinical application of biopsy in liver and pancreas for fat quantification purposes [4].

The medical imaging methods, including ultrasound, computed tomography (CT), and magnetic resonance imaging (MRI), are commonly used clinically for evaluating the fat content of liver and pancreas. Ultrasound examination relies on the operator's experience and lacks objective criteria, and the imaged field of view is also limited. Its diagnostic accuracy of mild and moderate fatty liver is poor and thus cannot be used for accurate visceral fat quantification [3, 5, 6]. CT is a semiquantitative method with good repeatability and has a high specificity for the diagnosis of moderate and severe liver fat deposits. However, there are also some limitations of applying CT for fat quantification. First, for monitoring the fat content changes for diabetes patients, CT is not suitable for a follow-up study due to ionizing radiation. Second, CT has a low diagnostic sensitivity to low-grade fatty liver. Third, CT value is sensitive to iron deposition in tissue, which may lead to an inaccurate measurement [7, 8].

With the development of MRI acquisition and reconstruction technology, the MR Dixon method is performed in routine clinical practice for water–fat separation. Previous studies proved that it can also be used for fat quantification noninvasively, the results of which consist with that of biopsy and have a higher accuracy and specificity than those of CT and ultrasound [9–11]. Engjom [12] demonstrated MR Dixon is superior than ultrasound in evaluating the fat content of pancreas, and the corresponding fat fraction (FF) result can be used as a marker of pancreatic secretion of failure. The purpose of this study was to quantify FF in liver and pancreas using MR Dixon and to further explore the differences in fat content between type 2 diabetes mellitus (T2DM) patients and healthy volunteers and the differences in fat content between obese T2DM patients and nonobese T2DM patients.

## 2. Materials and Methods

### 2.1. Patient Population

This study was approved by our institutional review board of Fujian Provincial Hospital (K2016-04-015) (Fuzhou, Fujian, China), and written informed consent was waived due to its retrospective nature. From May 2018 to May 2021, 118 T2DM patients (72 males and 46 females, age: 18–85 years old, average age 57.07, standard deviation 13.41) received treatment in our hospital (confirmed according to criteria for diagnosing diabetes WTO 1999), and 39 healthy volunteers (10 males and 29 females, age: 30–76 years old, average age 52.33, standard deviation 12.03) were enrolled in this study as control group. BMI, fasting blood glucose (FBG), high-density lipoprotein (HDL), low-density lipoprotein (LDL), triglyceride (TG), and cholesterol (CHOL) were acquired for all the patients and volunteers. The exclusion criteria were: (1) patients with type 1 diabetes or other special type diabetes, (2) alcohol intake: male ≥ 140 g/week or female ≥ 70 g/week [13], (3) patients confirmed with iron overload in liver or pancreas or received blood transfusion, (4) patients with chronic pancreatitis, pancreatic cancer, or patients with other diseases, which can cause fat deposition in pancreas, (5) a contraindication to MR imaging, (6) MR image quality is not sufficient for fat content calculation.

According to the criterion of the Chinese Diabetes Society, a BMI value higher than 25 was defined as obesity. All the subjects were divided into four groups, including Group 1: T2DM with BMI < 25 (37 males and 24 females, average age 59.28), Group 2: T2DM with BMI ≥ 25 (35 males and 22 females, average age 54.44), Group 3: control group with BMI < 25 (6 males and 22 females, average age 51.86), and Group 4: control group with BMI ≥ 25 (four males and seven females, average age 53.55).

### 2.2. MR Imaging Acquisition

All the MR exams were conducted on a 1.5T system (MAGNETOM Aera, SIEMENS Healthcare, Erlangen, Germany). Dual echo 3D VIBE sequence was performed for fat quantification purposes, and the detailed parameters were TR 6.46 ms, TE1/TE2 2.39/4.77 ms, FOV 380 × 380 mm, in-plane resolution 1.3 × 1.3 mm, slice thickness 3 mm and acquisition time 15 s. In order to reduce the motion artifacts, all patients were informed to hold breath during the data acquisition of the dual-echo VIBE sequence.

### 2.3. Measurement of FF of Liver and Pancreas

For liver, eight regions of interest (ROIs, with a size of 3 cm^2^) were depicted in left lateral lobe, left medial lobe, right anterior lobe, and right posterior lobe in the slice containing main portal vein and another slice below porta hepatis, respectively (Figure 1), by avoiding bile ducts, large vessels, lesions, the border of the liver and image artifacts. The average value of the eight ROIs was noted as the FF in whole liver (FFWL). In this study, we define FFWL < 5%, 5% ≤ FFWL <15%, 15% ≤ FFWL < 25%, and FFWL ≥ 25% as normal, mild, medium, and heavy fat content, respectively. Further, four ROIs (with a size of around 1.5 cm^2^) were located in head, neck, body, and tail of the pancreas (Figure 2), respectively, the average value of which was considered as the FF of whole pancreas (FFWP). The maximum diameters of the pancreas head, neck, body, and tail were recorded using the dual-echo VIBE images, and the average diameter of pancreas was also calculated using the four diameters mentioned earlier. All the abovementioned measurements were conducted on a commercial workstation (SIEMENS Healthcare, Erlangen, Germany).

### 2.4. Measurement of Abdominal Fat Area

The abdominal subcutaneous adipose area (SAT) and the visceral adipose tissue area (VAT) were measured using the FF image, which is 8 cm higher than the L4–L5 intervertebral space, by an open source software (ImageJ, https://imagej.nih.gov/ij/index.html). The total abdominal adipose tissue area (TAT) was calculated by adding SAT and VAT (Figure 3).

### 2.5. Statistical Analysis

The statistical analysis was performed with SPSS (version 22.0, SPSS inc., Chicago, IL, USA). The measured numerical data were presented as mean ± standard deviation. Intra- and intergroup comparison was made by employing independent sample *t*-test. The variance analysis was used to compare the fat content of the four study groups, and post hoc test was conducted with regard to the variables with significant differences in the four groups. Univariate logistic regression was used for all the variate, and then multivariate logistic regression was conducted with respect to the variate with statistical differences, so as to determine the independent predictor. *P* value < 0.05 was considered as statistically significant.

## 3. Results

### 3.1. Comparison between Group 1, Group 2, Group 3, and Group 4

#### 3.1.1. Comparison between Group 1 and Group 3

The values of FBG, TG, FFWL, FFWP, and the FF of the body and the tail of the pancreas and VAT in Group 1 were all higher than those in Group 3 (shown in Table 1). Univariate logistic regression indicated that, for patients and volunteers with BMI < 25, FBG (*B* = 1.59, Exp(*B*) = 4.94, *P* < 0.001), TG (*B* = 0.99, Exp(*B*) = 2.70, *P*=0.022), FFWL (*B* = 0.21, Exp(*B*) = 1.23, *P*=0.010), FFWP (*B* = 0.23, Exp(*B*) = 1.26, *P*=0.021), the FF of pancreas body (*B* = 1.60, Exp(*B*) = 1.17, *P*=0.048), the FF of pancreas tail (*B* = 0.22, Exp(*B*) = 1.24, *P*=0.018), and VAT (*B* = 0.01, Exp(*B*) = 1.01, *P*=0.020) are the risk factors for T2DM. Multivariate logistic regression indicated that FBG is the independent predictor for people with BMI < 25 (*B* = 1.59, Exp(*B*) = 4.94, *P* < 0.001).

#### 3.1.2. Comparison between Group 2 and Group 4

The values of FBG, TG, CHOL, FFWL, FFWP, the FF of the head of pancreas, and VAT in Group 2 are all higher than those in Group 4 (shown in Table 2). Through univariate logistic regression, it is indicated that, FBG (*B* = 2.30, Exp(*B*) = 10.03, *P*=0.002), HLD (*B* = −2.25, Exp(*B*) = 0.10, *P*=0.027), FFWL (*B* = 0.17, Exp(*B*) = 1.19, *P*=0.036), and VAT (*B* = 0.01, Exp(*B*) = 1.01, *P*=0.018) are the predictors for T2DM. The multivariate logistic regression analysis indicated that FBG (*B* = 3.52, Exp(*B*) = 33.84, *P*=0.028) and FFWP (*B* = 0.72, Exp(*B*) = 2.06, *P*=0.029) are the independent predictors for people with BMI ≥ 25.

#### 3.1.3. Comparison between Group 1 and Group 2

For T2DM patients, TG, CHOL, FFWL, FFWP, FF of the body and tail of pancreas, SAT, VAT, and TAT in Group 2 were all higher than those in Group 1, and HDL of Group 1 was lower than that of Group 2 (shown in Table 3).

#### 3.1.4. Comparison between Group 3 and Group 4

For control group, FPG, TG, FF of the tail of pancreas, SAT, and TAT in Group 4 (BMI ≥ 25) were all higher than those in Group 3 (BMI < 25) (shown in Table 4).

### 3.2. Comparison between T2DM Patients and Volunteers with Normal Liver Fat Content

As shown in Table 5, for subjects with normal liver fat content, FBG, FFWP, FF of pancreas, tail, and VAT of T2DM patients were higher than those of control volunteers, and HDL of T2DM patients were lower than that of control volunteers.

### 3.3. Comparison between T2DM Patients and Volunteers with Mild Liver Fat Content

As shown in Table 6, for subjects with mild liver fat content, FBG, FFWP, FF of pancreas, neck, and tail of T2DM patients were higher than those of control volunteers.

## 4. Discussion

With the continuous change in people's lifestyle and diet structure, unhealthy lifestyles, such as long-term intake of fat, lead to excessive accumulation of lipids in the human body. There is a close relationship between ectopic fat deposition and T2DM [1]. Such chronic noncommunicable disease needs early detection, early diagnosis, and early treatment, and thus, quantitative technique for tissue fat content is highly required in routine clinical practice.

Liver and pancreas biopsies are considered as the gold standard for fat quantification. However, due to its invasiveness, it is difficult to perform biopsies widely. Medical imaging modalities, like CT and ultrasound, can only be employed for qualitative diagnosis of tissue fat content; and CT exposes patients to ionizing radiation, which is not suitable for long-term follow-up treatment. All the limitations indicate that CT and ultrasound are not optimal for accurate tissue FF assessment.

Magnetic resonance spectroscopy (MRS) was also used for liver fat quantification in the previous paper. However, this study did not employ MRS to measure tissue fat content due to two reasons. First, high field homogeneity is required for MRS exams; not all MR scanners fulfill this requirement, especially the ones with large diameter. Second, current commercially available MRS technique in abdomen can only obtain signal of a single voxel, which cannot reflect fat deposition of the whole target tissue [2, 3, 5, 8]. MR Dixon technology is based on the principle of chemical shift between water and fat. By adjusting the echo time, in-phase and oppose-phase images are acquired within a single breath hold, which can be used for calculating the image of water or fat signals. A previous phantom study demonstrated that Dixon can provide accurate tissue fat content with reliable reproducibility. [14] Therefore, the present study used MR Dixon to derive tissue fat deposition, and further to analyze the fat content of T2DM patients and healthy subjects, and indicators of fat T2DM and normal T2DM patients.

For healthy people, fatty acids are stored in fat tissue in the form of triacylglycerol. When triacylglycerol exceeds the carrying capacity of adipose tissue, fat accumulates into nonfat tissue, such as liver and pancreas. The results of the present study show that the fat content of liver and pancreas of T2DM patients are higher than that of the control group. Previous studies have shown that fat deposition in liver causes insulin resistance, which may result in T2DM. Therefore, the presence of T2DM is highly related to the adipose deposition of liver [15, 16]. In Feng et al.'s paper [17], the liver FF of T2DM patients was higher than that of the normal subjects, which is consistent with our results. But no difference in pancreas fat content between T2DM and healthy volunteers was observed, which may be caused by their small sample size. At present, the relationship between pancreatic fat deposition and T2DM is not clear. Both Chai et al. [1] and Lu et al. [18] found that patients with T2DM had higher fat content in pancreas than that healthy people, which agreed with the results in the current study. Fatty pancreas has a higher proportion of T2DM than nonfatty pancreas group, indicating that fatty pancreas may have an association with T2DM [19]. This study demonstrated that the FF of pancreas head, body, and tail in T2DM patients are different from those of healthy volunteers. The univariate logistic regression analysis indicated that the adipose content in pancreas body and tail are the predictors of T2DM. Matsumoto et al. [20] reported that different parts of pancreas are generated from different embryologic pancreatic buds, resulting in the uneven fatty replacement of the pancreas. The posterior aspect of the head and the uncinate process of the pancreas lack adipose cells, but the anterior aspect of the head, the body, and the tail of the pancreas are sensitive to fat deposition, which agrees with the results of this study and may have a close relationship with T2DM.

Overweight or obesity is a risk factor for T2DM, but nonobese people may also suffer from diabetes. This study found that the FFWL, FFWP, and VAT are statistically different between NT2DM (T2DM, BMI < 25) and NCG (control group, BMI < 25). Through the analysis of single-factor logistic, the three indicators above are all influence factors in nonobese people with T2DM. Obesity could also cause dyslipidemia. In this study, for subjects with BMI ≥ 25, TG, and CHOL of T2DM patients were both higher than those of the corresponding volunteers; obese diabetic suffers from metabolism disorder, resulting in hyperlipidemia and other complications. Therefore, diabetic patients should pay attention to weight management, so as to prevent hyperlipidemia.

A previous study [21] showed that higher fasting and postprandial C-peptide levels and insulin resistance in nonobese patients with T2DM were independently associated with intra-abdominal adipose tissue volume. Free fatty acids and proinflammatory factors released by tissue fat can cause inflammatory reactions and insulin resistance in liver and pancreas after passing through the portal vein, leading to abnormality of blood sugar [22]. Comparing with subcutaneous fat, fat area in abdominal tissue has a higher correlation with blood glucose metabolism [23]. The findings in this study also demonstrates that VAT of T2DM patients is higher than that of the control group, and with the increase of tissue fat content, the occurrence of metabolic complications also increases [24, 25]. BMI, as the criterion of diagnosing obesity, can only assess the degree of obesity but not reflect the fat distribution in the human body. Therefore, it is necessary to not only pay attention to the BMI value but also to the tissue fat content when treating T2DM patients.

There are still some limitations in this study. First, the employed dual-echo Dixon sequence is sensitive to field inhomogeneity, which may generate phase error and further affect the accuracy of the FF calculation. On the other hand, ion deposition in the tissue, such as in liver, leads to the decrease of T2 ^*∗*^, which introduces calculation errors for fat quantification using dual-echo Dixon method. Such problem can be solved by using multi-echo Dixon technique. Accurate water, FF as well as T2 ^*∗*^ value can be derived simultaneously by fitting the acquired exponential decay curve. Previous researches [26, 27] showed that the liver fat content generated by a six-echo Dixon sequence had a high association with that obtained by MRS and biopsy, respectively. However, such advanced sequence is not equipped in the employed scanner in this study and will be used for analyzing the tissue adipose content of T2DM patients in our future plan.

## 5. Conclusion

The evaluation of tissue FF plays an important role in the development of diabetes. MR Dixon technique has the clinical potential to quantify the adipose content noninvasively, which will be helpful for T2DM patients.

## Figures and Tables

**Figure 1:** For liver, eight regions of interest (ROIs) were depicted in left lateral lobe, left medial lobe, right anterior lobe, and right posterior lobe in the slice contains the main portal vein (a) and two slices below porta hepatis (b), respectively.

**Figure 2:** ROIs (with a size of around 1.5 cm^2^) were located in head (a), neck (b), body (c), and tail (d) of the pancreas, respectively.

**Figure 3:** The abdominal subcutaneous adipose area (SAT) (a) and the visceral adipose tissue area (VAT) (b) were measured using the FF image, which is 8 cm higher than the L4–L5 intervertebral space, by an open-source software (ImageJ, https://imagej.nih.gov/ij/index.html).

**Table 1:** Comparison of tissue FF and clinical indicators between Group 1 and Group 3.

	Group 3	Group 1	*P*
FBG (mmol/l)	4.93 ± 0.66	8.83 ± 3.47	<0.001
HDL (mmol/l)	1.50 ± 0.86	1.19 ± 0.44	0.032
LDL (mmol/l)	2.76 ± 0.97	3.03 ± 0.93	0.239
TG (mmol/l)	1.09 ± 0.49	1.75 ± 1.41	0.002
CHOL (mmol/l)	4.35 ± 1.09	4.73 ± 1.10	0.149
FFWL (%)	4.17 ± 2.52	7.86 ± 5.95	<0.001
FF of pancreas head (%)	6.81 ± 4.69	7.63 ± 3.84	0.381
FF of pancreas neck (%)	7.52 ± 3.45	9.11 ± 3.86	0.064
FF of pancreas body (%)	7.12 ± 2.67	8.88 ± 4.10	0.040
FF of pancreas tail (%)	6.91 ± 2.11	9.10 ± 4.47	0.002
FFWP (%)	7.09 ± 2.60	8.68 ± 3.00	0.012
Average diameter of pancreas (cm)	1.64 ± 0.29	1.84 ± 1.79	0.565
SAT (cm^2^)	91.46 ± 39.48	88.05 ± 39.44	0.704
VAT (cm^2^)	69.36 ± 54.77	97.13 ± 47.74	0.016
TAT (cm^2^)	160.82 ± 81.15	185.19 ± 61.41	0.117

**Table 2:** Comparison of tissue FF and clinical indicators between Group 2 and Group 4.

	Group 4	Group 2	*P*
FBG (mmol/l)	5.45 ± 0.60	9.06 ± 2.75	<0.001
HDL (mmol/l)	1.24 ± 0.48	0.98 ± 0.27	0.121
LDL (mmol/l)	3.17 ± 0.77	3.10 ± 0.98	0.821
TG (mmol/l)	1.79 ± 0.78	5.13 ± 7.15	0.002
CHOL (mmol/l)	4.79 ± 0.56	5.65 ± 2.13	0.014
FFWL (%)	6.04 ± 3.63	13.85 ± 9.18	<0.001
FF of pancreas head (%)	6.50 ± 2.15	8.69 ± 4.69	0.022
FF of pancreas neck (%)	7.86 ± 2.47	9.07 ± 5.95	0.512
FF of pancreas body (%)	9.00 ± 3.54	10.83 ± 4.81	0.237
FF of pancreas tail (%)	8.94 ± 2.25	11.19 ± 5.19	0.165
FFWP (%)	8.08 ± 1.95	9.95 ± 3.87	0.025
Average diameter of pancreas (cm)	1.67 ± 0.35	2.18 ± 1.86	0.375
SAT (cm^2^)	137.96 ± 84.95	124.72 ± 67.74	0.573
VAT (cm^2^)	108.03 ± 51.75	172.22 ± 77.42	0.011
TAT (cm^2^)	245.99 ± 119.63	296.94 ± 116.10	0.192

**Table 3:** Comparison of tissue FF and clinical indicators between Group 1 and Group 2.

	Group 1	Group 2	*P*
FBG (mmol/l)	8.83 ± 3.47	9.06 ± 2.75	0.691
HDL (mmol/l)	1.19 ± 0.44	0.98 ± 0.27	0.001
LDL (mmol/l)	3.03 ± 0.93	3.10 ± 0.98	0.678
TG (mmol/l)	1.75 ± 1.41	5.13 ± 7.15	0.001
CHOL (mmol/l)	4.73 ± 1.10	5.65 ± 2.13	0.006
FFWL (%)	7.86 ± 5.95	13.85 ± 9.18	<0.001
FF of pancreas head (%)	7.63 ± 3.84	8.69 ± 4.69	0.177
FF of pancreas neck (%)	9.11 ± 3.86	9.07 ± 5.95	0.965
FF of pancreas body (%)	8.88 ± 4.10	10.83 ± 4.81	0.019
FF of pancreas tail (%)	9.10 ± 4.47	11.19 ± 5.19	0.021
FFWP (%)	8.68 ± 3.00	9.95 ± 3.87	0.048
Average diameter of pancreas (cm)	1.84 ± 1.79	2.18 ± 1.86	0.318
SAT (cm^2^)	88.05 ± 39.44	124.72 ± 67.74	0.001
VAT (cm^2^)	97.13 ± 47.74	172.22 ± 77.42	<0.001
TAT (cm^2^)	185.19 ± 61.41	296.94 ± 116.10	<0.001

**Table 4:** Comparison of tissue FF and clinical indicators between Group 3 and Group 4.

	Group 3	Group 4	*P*
FPG (mmol/l)	4.93 ± 0.66	5.45 ± 0.60	0.031
HDL (mmol/l)	1.50 ± 0.86	1.24 ± 0.48	0.385
LDL (mmol/l)	2.76 ± 0.97	3.17 ± 0.77	0.223
TG (mmol/l)	1.09 ± 0.49	1.79 ± 0.78	0.002
CHLO (mmol/l)	4.35 ± 1.09	4.79 ± 0.56	0.120
FF of pancreas head (%)	6.81 ± 4.69	6.50 ± 2.15	0.838
FF of pancreas neck (%)	7.52 ± 3.45	7.86 ± 2.47	0.767
FF of pancreas body (%)	7.12 ± 2.67	9.00 ± 3.54	0.079
FF of pancreas tail (%)	6.91 ± 2.11	8.94 ± 2.25	0.012
FFWP (%)	7.09 ± 2.60	8.08 ± 1.95	0.264
Average diameter of pancreas (cm)	1.64 ± 0.29	1.67 ± 0.35	0.799
SAT (cm^2^)	91.46 ± 39.48	137.96 ± 84.95	0.024
VAT (cm^2^)	69.36 ± 54.77	108.03 ± 51.75	0.051
TAT (cm^2^)	160.82 ± 81.15	245.99 ± 119.63	0.014

**Table 5:** Comparison between T2DM patients and volunteers with normal liver fat content.

	Volunteers	T2DM patients	*P*
FBG (mmol/l)	5.12 ± 0.68	8.55 ± 3.48	<0.001
HDL (mmol/l)	1.54 ± 0.83	1.23 ± 0.43	0.049
LDL (mmol/l)	2.86 ± 0.91	2.90 ± 0.91	0.859
TG (mmol/l)	1.25 ± 0.66	1.36 ± 0.77	0.549
CHOL (mmol/l)	4.53 ± 1.00	4.48 ± 0.98	0.844
FF of pancreas head (%)	6.36 ± 3.61	7.83 ± 4.11	0.120
FF of pancreas neck (%)	7.49 ± 3.05	8.35 ± 4.53	0.373
FF of pancreas body (%)	7.30 ± 3.19	8.08 ± 3.40	0.327
FF of pancreas tail (%)	7.41 ± 2.28	9.83 ± 5.29	0.009
FFWP (%)	7.14 ± 2.38	8.52 ± 3.00	0.040
Average diameter of pancreas (cm)	1.64 ± 0.30	1.64 ± 0.31	0.906
SAT (cm^2^)	93.35 ± 45.30	91.63 ± 44.93	0.874
VAT (cm^2^)	65.62 ± 48.22	100.58 ± 63.65	0.014
TAT (cm^2^)	158.97 ± 82.63	192.21 ± 81.09	0.093

**Table 6:** Comparison between T2DM patients and volunteers with mild liver fat content.

	Volunteers	T2DM patients	*P*
FBG (mmol/l)	5.02 ± 0.70	9.20 ± 3.19	<0.001
HDL (mmol/l)	1.09 ± 0.44	0.99 ± 0.36	0.490
LDL (mmol/l)	2.97 ± 0.99	2.97 ± 1.08	0.999
TG (mmol/l)	1.49 ± 0.69	3.75 ± 6.38	0.299
CHOL (mmol/l)	4.35 ± 0.92	5.06 ± 1.94	0.296
FF of pancreas head (%)	7.77 ± 5.40	9.69 ± 4.04	0.227
FF of pancreas neck (%)	7.99 ± 3.67	11.46 ± 4.22	0.024
FF of pancreas body (%)	8.68 ± 2.26	11.26 ± 5.67	0.169
FF of pancreas tail (%)	7.69 ± 2.50	11.85 ± 6.19	0.046
FFWP (%)	8.03 ± 2.66	11.07 ± 3.89	0.026
Average diameter of pancreas (cm)	1.70 ± 0.33	1.68 ± 0.30	0.846
SAT (cm^2^)	137.15 ± 81.38	109.23 ± 58.77	0.234
VAT (cm^2^)	122.73 ± 57.97	140.35 ± 62.39	0.430
TAT (cm^2^)	259.88 ± 111.21	249.58 ± 89.67	0.764

## Data Availability

The datasets analyzed during the current study are available from the corresponding author upon reasonable request. All data generated or analyzed during this study are included in this published article.
